# 3D M-Net: Object-Specific 3D Segmentation Network Based on a Single Projection

**DOI:** 10.1155/2021/5852595

**Published:** 2021-07-12

**Authors:** Xuan Li, Sukai Wang, Xiaodong Niu, Liming Wang, Ping Chen

**Affiliations:** State Key Lab for Electronic Testing Technology, North University of China, Taiyuan 030051, China

## Abstract

The internal assembly correctness of industrial products directly affects their performance and service life. Industrial products are usually protected by opaque housing, so most internal detection methods are based on X-rays. Since the dense structural features of industrial products, it is challenging to detect the occluded parts only from projections. Limited by the data acquisition and reconstruction speeds, CT-based detection methods do not achieve real-time detection. To solve the above problems, we design an end-to-end single-projection 3D segmentation network. For a specific product, the network adopts a single projection as input to segment product components and output 3D segmentation results. In this study, the feasibility of the network was verified against data containing several typical assembly errors. The qualitative and quantitative results reveal that the segmentation results can meet industrial assembly real-time detection requirements and exhibit high robustness to noise and component occlusion.

## 1. Introduction

In the industrial production process, real-time assembly detection is an essential link [1]. Especially for critical disposable products (such as fuses, solid rocket motors, and airbags), conventional functional testing destroys the product structure. Due to the particularity of this kind of product, abnormal assembly inevitably causes notable safety hazards and property losses, so these products must be detected one at a time before being put into use. Therefore, a real-time automatic assembly detection method that can match the production rhythm is highly important to improve production efficiency and product reliability.

Since X-rays can obtain internal information, this technology is widely applied in internal abnormality detection. To ensure the detection speed, a series of internal abnormality detection methods based on a single projection has been widely implemented in different fields, such as the security field [2–5] and the aerospace field [6–8]. These methods achieve rapid detection via the direct extraction of features from projections. However, in regard to the assembly detection of industrial products, these kinds of single-projection methods are susceptible to component occlusion, thereby reducing the accuracy. The main reason is that industrial products possess complex structures, and the distribution of internal components is compact, so component occlusion is inevitable. Furthermore, projections contain integral information of all the components passed by the ray path. It is difficult to separate the information contribution of the different components. An effective way to avoid occlusion is to apply computed tomography (CT) algorithms. The 3D model of the product can provide richer structural information for detection while avoiding the influence of occlusion. However, the CT reconstruction algorithm requires complete projection data and consumes much time. Limited by the projection data acquisition speed and reconstruction speed, the CT reconstruction approach does not meet the needs of real-time detection.

Researchers have introduced convolutional neural networks (CNNs) [9] based on deep learning [10] in the field of X-ray 3D reconstruction and proposed a series of single-projection 3D reconstruction algorithms for specific targets. Henzler et al. [11] used the encoder-decoder network [12] to predict a low-resolution 3D model and fused the result with the projection to improve the resolution, thus achieving single-projection reconstruction of the mammalian skull. Shen et al. [13] designed an automatic encoder network with an embedded conversion module and used the feature representation across dimensions to realize reconstruction of specific patients based on ultrasparse projection data. On this basis, Lei et al. [14] introduced generative adversarial networks (GANs) [15], using adversarial supervision to improve the realism of generated 3D images relative to ground truth images. Wang et al. [16] employed multiorgan template selection and smooth free-form deformation (FFD) strategies to generate high-quality manifold meshing models of organs. Based on the U-Net [17], Vlontzos et al. [18] proposed the 2D to 3D U-Net, which realizes 3D volume generation of the target organ based on a single projection. Compared to the traditional CT reconstruction algorithms, the above algorithms do not reconstruct 3D volumes by solving the mathematical inversion but rely on structural features extracted from the projection for reconstruction. By combining the structural priors implied in the dataset of a specific target, the 3D structure of the reconstruction result is constrained, thereby achieving a single-projection reconstruction of the specific target. These single-projection reconstruction algorithms highly reduce the data acquisition time, thus facilitating real-time detection based on 3D data.

The purpose of assembly detection is to determine the position and posture of different product components. Through segmentation of the internal components of a given product, the results of the segmentation algorithm can be applied to accurately determine the position and posture of the components. Since Long et al. [19] first applied fully convolutional networks (FCNs) to image segmentation, semantic image segmentation based on CNNs has become a research area of heightened interest, and many breakthroughs have been achieved. Researchers have successively proposed DeconvNet [20], SegNet [21], U-Net, LinkNet [22], DeepLab [23], PSPNet [24], and other image segmentation networks based on CNNs. These semantic image segmentation networks can be summarized as encoder-decoder networks, where the encoder is adopted for image feature extraction, and the decoder is employed to map the learned semantic features onto the pixel space to obtain the probabilistic classification of the different pixels. These algorithms are widely adopted in the medical field and have achieved many results [25–27]. However, these works segment the target from 2D slices, only consider 2D features in the cross section and ignore 3D features. Regarding assembly detection, industrial products contain many components with similar cross-sectional features but different 3D structures. It is difficult to accomplish an accurate distinction only via 2D segmentation of the cross section. Aiming at the semantic segmentation of 3D images, Milletari et al. [28] proposed a fully convolutional 3D segmentation network (V-Net) to directly segment the 3D volume and designed the Dice loss function to train the network. Yang et al. [29] introduced a pyramid pooling module into a 3D convolutional network and adopted a combination of global and local features for more accurate voxel prediction. In contrast to the above single-target segmentation algorithms, Gibson et al. [30] designed a dense FCN (Dense V-Net) for multicategory 3D segmentation.

In terms of assembly detection, whether the assembly is correct or not, the product exhibits a similar structure, with only partial differences. Based on this characteristic, by combining the single-projection reconstruction algorithm and the 3D segmentation algorithm, we proposed an end-to-end X-ray single-projection 3D segmentation network for specific products. The network adopts a single projection of any view as input and performs segmentation of different components under the same perspective. The proposed approach first generates asymmetric mappings with a deep encoder-decoder network under the constraints of a specific dataset, thereby adaptively extracting features from 2D projections and mapping them onto the 3D space domain. In the mapping process, by postponing cross-dimensional feature transformation and applying 2D convolution instead of 3D convolution for upsampling, the feature processing flow is optimized to reduce the calculations. Furthermore, a mixed loss function comprising Dice and cross-entropy terms is applied to solve the data imbalance issue. Compared to CT-based detection methods, the application of this network in assembly detection can reduce the data acquisition time and achieve real-time detection. Furthermore, this network can help to simplify imaging hardware and improve radiation utilization, thus reducing detection costs. To our knowledge, this is the first article to propose a single-projection 3D segmentation network.

## 2. Methods

### 2.1. Principle

The essence of semantic image segmentation algorithms is the pixelwise classification algorithm, which can be broadly regarded as involving the two stages of feature extraction and feature mapping. At the feature extraction stage, cascaded convolutional layers are used for feature extraction, usually accompanied by downsampling to reduce the dimensionality of features and finally form the semantic features of the image. At the feature mapping stage, upsampling is performed to map the learned discriminative features onto a high-resolution pixel space. Different networks add various feature transfer mechanisms (skip connection [17], pyramid pooling [24], etc.) to increase the information and accuracy of mapping. Finally, a probability vector is constructed for each pixel, and pixelwise classification is achieved via the prediction of pixels belonging to the different targets. Most image segmentation networks (such as FCNs [19], SegNet [21], and U-Net [17]) follow this process and have achieved great segmentation results. The projections and the reconstruction results should share semantic features, as they represent the same object [13]. Based on this consideration, previous works on single-projection reconstruction [11, 13, 14] have verified that, under the strict constraint condition that the structure of specific targets is similar, the 2D features containing local differences extracted from projections can be mapped onto 3D features and correctly expressed in the constructed 3D output. This study combines this idea with the semantic image segmentation algorithm to achieve 3D segmentation of specific targets based on a single projection. The following three problems need to be solved:

1. Computational cost of 3D feature processing: It is necessary to improve the efficiency of 3D feature processing to realize real-time segmentation under existing hardware resources.
2. Cross-dimensional manifold mapping: It is necessary to map the 2D features of the projection image onto the 3D structural features of the object in order to construct the probability vector output of the 3D voxels.
3. Data imbalance: It is necessary to solve the problem of inconsistent training efficiency for different segmentation targets due to volume differences.

Taking these three problems as clues, the following content of this section introduces the network architecture and loss function.

### 2.2. Network Architecture

The proposed network can be regarded as an extension of the encoder-decoder network model [12] and follows the process of feature extraction and feature mapping. As shown in Figure 1, the encoder network comprises four residual convolution blocks and five downsampling blocks. The residual convolution blocks extract 2D features from the input projections and gradually increase feature channels to 512. The downsampling blocks gradually reduce the spatial size of the input feature map to 8 × 8 and keep the number of feature channels unchanged so that convert high-dimensional features into low-dimensional embedded semantic representations. The decoder network consists of five upsampling blocks, a feature transformation model, and three 3D convolution blocks. The upsampling blocks restore the low-dimensional features and gradually increase the spatial size of the feature maps to the target size (256 × 256). The feature transformation model transforms the high-dimensional feature representation across dimensions for the subsequent generation of the probability vector. Then, the number of channels of the 3D features is gradually increased through the 3D convolution blocks to ensure that the output is of the same size as that of the target probability vector (256 × 256 × 256). Finally, the probability vector of each voxel is obtained through the softmax layer. Refer to section 2.5 for detailed network parameter settings.

### 2.3. Improve the Efficiency of Feature Processing

The 3D convolution process can maintain the spatial association of features and control the size of the output feature, so it is an essential operation in 3D segmentation. However, 3D convolution is associated with a large number of parameters and computations, occupying a large amount of memory. Under the existing hardware resources, this limits the resolution and speed of the segmentation algorithm. This problem is common in 3D segmentation networks and is usually solved by improving hardware utilization and optimizing the algorithm's computing efficiency. For example, literature [30] achieved high-resolution 3D segmentation through memory-efficient dropout and feature reuse.

To improve the feature processing efficiency to realize real-time 3D segmentation of industrial products, we postponed feature cross-dimensional mapping and 3D convolution in the decoder network and adopted the same technique as reported in the literature [11], applying 2D convolution instead of 3D convolution for upsampling (as shown by the green arrow in Figure 1). 3D convolution is only employed in probability vector construction from 3D features (as shown by the red arrow in Figure 1). Specifically, in the 3D segmentation network, feature mapping in the decoder network is usually implemented via 3D convolution. The computation is mainly concentrated on upsampling. To improve the computational efficiency, we encode depth information into the channel dimension and apply 2D convolution instead of 3D convolution for upsampling, which highly reduces the number of parameters and computation. Since downsampling and upsampling comprise convolution processes with the same dimensions, skip connections similar to those in the U-Net [17] can be used in the network (shown by the dotted arrow in Figure 1). This can provide more detailed information for the feature mapping process, which is helpful for the segmentation of tiny structures. In the process of downsampling and upsampling, the feature channel is fixed to twice the spatial resolution, i.e., 2 × 256 = 512. The structure of the downsampling and upsampling blocks and skip connections is shown in Figures 2(b) and 2(c), respectively. In addition, because of the notable depth of the network, in all 2D convolution operations (residual convolution blocks, downsampling blocks, and upsampling blocks), we adopt the residual learning scheme [31] to improve the training efficiency and avoid gradient disappearance, as shown in Figure 2(a).

### 2.4. Cross-Dimensional Feature Mapping

In the process of downsampling and upsampling, depth information is encoded in the channel dimension of the feature. This process can be regarded as a process involving the extraction and fusion of depth and structural information. To bridge the upsampling blocks and subsequent 3D convolution blocks, we designed a feature transformation model to decode depth information and realize cross-dimensional mapping. As shown in Figure 2(d), through the convolution operation with a kernel size of 1 × 1 and rectified linear unit (ReLU) activation, the 2D convolutional layer learns the transformation of all 2D features and reorganizes the depth information implicit in the channel dimension. Then, the feature map is reshaped from 256 × 256 × 512 to 256 × 256 × 256 × 2. In this manner, the 2D features are transformed across dimensions for the subsequent generation of the probability vector. Next, we apply the 3D convolution operation with a kernel size of 1 × 1 × 1 and a stride of 1 × 1 × 1 to learn the transformations among all 3D features and maintain the feature size unchanged. The feature transformation model connects the 2D and 3D feature domains and maps the 2D features with hidden depth information into 3D features.

### 2.5. Details of the Network Structure and Parameters

The parameter settings of the entire network are summarized in Tables 1 and 2. The encoder network and the upsampling process in the decoder network comprise residual blocks. Each residual block comprises two sets of 3 × 3 2D convolutional layers, batch norm layers, and ReLU activation functions. A residual path is added between the input and the second ReLU through a 1 × 1 convolution layer. As input, the projection first performs 2D feature extraction through four residual blocks, thereby maintaining the spatial size fixed and gradually expanding the channels to 512. The downsampling block comprises two residual blocks and a 2 × 2 max-pooling layer. Five downsampling blocks constitute the compression path of the feature stream. Through downsampling, a low-resolution feature with a large receptive field is gradually established, with a size of 8 × 8 × 512. The upsampling block comprises a 2D deconvolution layer (with a kernel size of 3 × 3 and a stride of 2 × 2) and two residual blocks. Five upsampling blocks constitute the extension path of the feature stream. Through upsampling, the spatial size of the feature maps is gradually restored to 256 × 256 × 512, which expands the spatial support of the lower-resolution feature maps. Via upsampling and downsampling, the depth information encoded in the channel dimension is integrated and reorganized. Between the upsampling and downsampling blocks of the same level, a path of feature flow transfer is added through a skip connection. In the skip connection, the feature maps from the downsampling block and previous upsampling block are first concatenated and then merged through a 1×1 2D convolution operation to ensure that the number of channels remains fixed at 512. After passing through the feature transformation module, the 2D features with hidden depth information are transformed into 3D features. Next, three 3D convolution blocks are employed to reorganize the structural features and expand the channels. Each 3D convolution block comprises a 3 × 3 × 3 3D convolution layer, a batch norm layer, and a ReLU activation function. Finally, the network output is adjusted to a suitable size via 1 × 1 × 1 3D convolution and transformed into a probability vector by the softmax layer.

### 2.6. Loss Function

Due to differences in the sample number among the various segmentation targets, the network often ignores categories containing fewer samples, which in turn affects the segmentation effect of these categories [32]. In terms of the 3D segmentation of components in industrial products, the data imbalance issue is mainly reflected in the number of voxels. The voxel number of the components of different sizes often differs by several orders of magnitude. This kind of difference cannot be balanced through data enhancement, so in this study, we address this problem via loss function optimization.

The output of the proposed network is processed by the softmax layer for multiclassification, and the probability of each voxel belonging to the background or a certain component is calculated. To optimize the segmentation performance of the network, the accuracy of the predicted probability over the ground truth must be evaluated via calculating loss function. As a common loss function applied in segmentation, the Dice loss function [28] measures the accuracy of prediction by calculating the ratio between the intersection and union of the segmentation and ground truth regions. The Dice loss between the predicted probability *P* and ground truth *R* can be expressed as follows:

(1) $$\begin{array}{c} {ℒ}_{\text{Dice}}\left(P,R\right)=1-\frac{1}{M}\sum_{i=1}^{M}\frac{2\sum_{j=1}^{N}p_{i,j}r_{i,j}+\varepsilon }{\sum_{j=1}^{N}p_{i,j}^{2}+\sum_{j=1}^{N}r_{i,j}^{2}+\varepsilon }. \end{array}$$

where *M* is the number of categories in the probability vector, and each category represents a kind of component or background (the background is set to category 0). Moreover, *N* is the number of voxels, *p*_*i,j*_ and *r*_*i,j*_ denote the probability that the *j*^*th*^ voxel belongs to the *i*^*th*^ category in the predicted probability and the ground truth, respectively. And *ε* is applied to prevent the denominator from equalling 0, which is set to 10^−10^ in this study. The Dice loss balances the voxel number of the different categories through the square term in the denominator. However, due to the complex gradient form of the Dice loss, gradient saturation occurs in the training process, which often leads to training instability. To solve this problem, we added a weighted cross-entropy (WCE) term to the Dice loss. The WCE loss is defined as follows:

(2) $$\begin{array}{c} {ℒ}_{WCE}=\sum_{i=1}^{M}\left(\sum_{j=1}^{N}\omega_{i}r_{i,j}\log\left(p_{i,j}\right)\right),\\ \omega_{i}=\frac{1}{\sum_{j=1}^{N}r_{i,j}+\varepsilon }, \end{array}$$

where *ω*_*i*_ is the weight of the *i*^*th*^ category, which is used to penalize the gradient contribution of the large-size component in training. Therefore, the mixed loss is defined as follows:

(3) $$\begin{array}{c} ℒ=\alpha {ℒ}_{\text{Dice}}+\left(1-\alpha \right){ℒ}_{\text{WCE}}. \end{array}$$

where *α* balances the Dice and the WCE terms, which is set to 0.5.

### 2.7. Implementation Details

The network is implemented using the Tensorflow framework and optimized with the Adam optimizer at an initial learning rate of 10^−4^ and a minibatch size of 5. In the training process, we evaluate the model on the validation set and gradually reduce the learning rate from 10^−4^ to 10^−6^. The training and testing of the network are carried out on a workstation with an E5-2620 CPU, 32 GB of RAM, and a TITAN RTX GPU.

## 3. Material

Taking a fuse as the detection target, we perform data acquisition. Under the best imaging conditions, we acquire 1080 projections of the fuse at equal angular intervals on the YXLON FF20 CT system with tube voltage 160 kV and current 40 *μ*A and then adopt the FDK algorithm for reconstruction. Next, regarding the 14 critical fuse components, the reconstructed 3D image was manually segmented. Specifically, each reconstructed slice was segmented with the watershed algorithm involving artificial participation, and all the segmented slices were then combined into a 3D segmented image as the ground truth data for training the network. Since the perspective of the reconstruction result depends on the order of the projections, we reordered the projections before reconstruction so that the components attained the same spatial distribution in the reconstruction results. In addition, as the input of the network, the projections were resized into 256 × 256 and normalized to [0, 1]. For the convenience of description, we numbered the 14 critical components, as shown in Figure 3.

Regarding the most error-prone striker and spring, according to typical assembly errors (posture error, position error, and omission), we set a total of six different assembly situations, as shown in Figure 4. For each situation, 12 sets of data were generated through the abovementioned data acquisition process. Before acquiring each set of data, the fuse has been reassembled. Ten sets of data were used for training. Moreover, to control the size of the training dataset, we randomly selected half of them as the training dataset, containing 32400 samples. The rest two sets were reserved for validating and testing, each containing 6480 samples.

## 4. Experiment Results and Discussion

### 4.1. Segmentation Results of the Proposed Network

We evaluate the segmentation performance of our network on the test dataset and randomly select a sample from each assembly situation for display. Figure 4 shows the 3D rendering of the segmentation results. To avoid occlusion, the results are shown as anatomical diagrams. In addition, we randomly select four slices from the segmentation results to compare the segmented foreground regions, as shown in Figure 5. The yellow, red, and green areas represent the ground truth, predicted segmentation, and overlap area, respectively. To increase the prominence of the difference, we display magnified views of partial areas. Furthermore, we adopt four metrics for quantitative analysis of the network segmentation results, namely, the Dice similarity coefficient (DSC), Jaccard similarity coefficient (JSC), positive prediction value (PPV), and sensitivity (SEN). These metrics are defined as follows:

(4) $$\begin{array}{c} \text{DSC}=\frac{2\left\|V_{gt}\cap V_{pd}\right\|}{\left\|V_{gt}\right\|+\left\|V_{pd}\right\|},\\ \text{JSC}=\frac{\left\|V_{gt}\cap V_{pd}\right\|}{\left\|V_{gt}\cup V_{pd}\right\|},\\ \text{PPV}=\frac{\left\|V_{gt}\cap V_{pd}\right\|}{\left\|V_{pd}\right\|},\\ \text{SEN}=\frac{\left\|V_{gt}\cap V_{pd}\right\|}{\left\|V_{gt}\right\|}, \end{array}$$

where *V*_*gt*_ and *V*_*pd*_ denote the ground truth and predicted segmentation voxels, respectively. The quantitative results of the different component segmentations are summarized in Table 3.

The qualitative and quantitative analysis results indicate that the difference between the segmentation result of the network and the manual segmentation result is very small. The differences are mainly concentrated along the edge of the components and include mispredicted scattered points. The segmentation results fully reflect the assembly situation of the fuse. The advantage of the network is that the use of projections from any angle as the input can reduce the dependence on mechanical equipment, which helps simplify the imaging system and reduce the cost of detection. In addition, the segmentation results output by the network are generated in the same perspective, which allows the position and posture information obtained from the segmentation results to be directly used to infer the assembly situation without any coordinate transformation.

### 4.2. Comparison to General 3D Segmentation Networks

To our knowledge, there is no 3D segmentation algorithm based on a single projection. Therefore, we compare our network to general segmentation algorithms based on 3D images. U-Net [17] and V-Net [28] are the baseline architectures for 2D and 3D image segmentation, respectively, which have been widely applied and adapted. Therefore, V-Net and 3D U-Net [33] (a 3D variant of U-Net) are selected as candidates for comparison. Since the original V-Net and 3D U-Net are designed for binary segmentation, we extend their loss functions to support multiclass data. Applying the CT reconstruction result and artificial segmentation result as the input and ground truth data, we train the V-Net and 3D U-Net on the training dataset and then test these networks on the test dataset. The qualitative and quantitative results of the different algorithms are shown in Figures 6 and 7 and Table 4.

The comparison reveals that the difference between the segmentation results obtained with the proposed network and the general 3D segmentation networks is extremely small. The performance of the proposed network almost reaches the level of the general 3D segmentation algorithms. It should be emphasized that the proposed network uses a single projection as the input for 3D segmentation, and a single segmentation requires approximately 0.2 seconds. Applying this network to industrial product assembly detection can greatly reduce the time required for data acquisition and 3D reconstruction and achieve real-time detection, which is of great significance for industrial products with a high production speed and huge production.

### 4.3. Segmentation Results with Noise

Quantum fluctuation noise in radiography obeys the Poisson distribution. Therefore, Poisson noise is added to the projections for analysis to illustrate the robustness of our network to noise. Noise addition is according to the following formula:

(5) $$\begin{array}{c} P_{i}∼\text{Possion}\left\{b_{0}e^{-l_{i}}\right\}, \end{array}$$

where *P*_*i*_ is the detector measurement along the *i*^*th*^ ray, *b*_*0*_ is the blank scan factor, and *l*_*i*_ is the line integral of the attenuation coefficients along the *i*^*th*^ ray. The Poisson noise level can be adjusted by setting the blank scan factor *b*_*0*_. In this study, *b*_*0*_ is varied from 1 × 10^6^ to 1 × 10^3^. During the decrease of *b*_*0*_, several segmentation results with notable changes are shown in Figure 8. The performance metrics of the segmentation results are summarized in Table 5.

Before *b*_*0*_ decreases to 1 × 10^5^, the segmentation performance of the network remains relatively stable. When the noise level is worse than 1 × 10^4^, the components in the segmentation results start to exhibit adhesion and the number of scattered points increases. When the noise level further deteriorates to 4 × 10^3^, part of the information in the projection is masked by the noise. In the segmentation results, certain components are structurally missing, and the number of scattered points further increases. The results demonstrate that when *b*_*0*_ is greater than 1 × 10^5^, the network effectively suppresses noise, and the segmentation results completely and accurately reflect the position, structure, and posture information of each component. The proposed network remains robust to a relatively broad range of noise levels.

### 4.4. Segmentation Results with Occlusion

We selected samples in different occlusion cases for comparison.  Figure 9 shows the segmentation results in the three occlusion cases and the grayscale level profiles extracted along the dashed red line.

In the projections and the grayscale level profiles, it is difficult to determine whether the striker exists in cases 2 and 3 with the naked eye. Comparing the former two samples demonstrates that the network can use projections from different angles for segmentation and can completely segment the occluded component. Comparing the latter two samples reveals that the network can perform correct segmentation in the different assembly situations with similar projections. Therefore, the proposed network achieves high robustness to occlusion. In assembly detection, the network can effectively avoid the influence caused by component occlusion.

### 4.5. Segmentation Results with Untrained Assembly Errors

In order to further verify the effectiveness of the proposed network, we set up two additional assembly errors for the spring and the striker (the striker missed with the spring stuck upside, and the spring missed with the striker stuck upside) and acquire the data under these two wrong assembly conditions for testing. The segmentation results are shown in Figure 10 and Table 6.

The results indicate that for untrained assembly errors, the network can also correctly extract the features of each component and perform correct segmentation. Compared with the trained data, there is no noticeable difference in the performance metrics of the segmentation results. Therefore, for the assembly errors of the striker and the spring, the segmentation results can be applied to detect effectively.

## 5. Conclusion

In this study, we proposed a multiclass 3D segmentation network based on a single X-ray projection by combining the single-projection reconstruction algorithm and the semantic image segmentation algorithm. Adopting a single projection as the input, the network can segment different targets within a specific object and can output 3D segmentation results. The experimental results indicate that the segmentation results of the network completely reflect the position, structure, and posture information of the different internal targets, and the segmentation performance for the specific objects is close to that of the 3D semantic image segmentation network. In addition, the network achieves high robustness to noise and component occlusion. The advantage of implementing the network in assembly detection is that it takes a single projection to perform 3D segmentation, which can improve the ray utilization rate and detection efficiency, thereby realizing real-time detection. Furthermore, the network is suitable for projections from different angles, which can simplify the imaging system and help reduce detection costs.

In the application process, the network can be directly deployed in digital radiography detection systems without any additional machinery or imaging equipment. However, the network has certain drawbacks and limitations. First, in contrast to the general semantic image segmentation algorithm, the network performs segmentation of specific objects, which suggests that changing the detection products requires network retraining. Second, the network relies on complete training data, which means that it needs to acquire data of different assembly situations for training.

To solve the problem whereby training data are difficult to obtain, in future work, we plan to conduct research on simulation data synthesis to reduce the difficulty and time cost of training data acquisition.

## Figures and Tables

**Figure 1:** Schematic of the network architecture. The encoder network consists of residual convolution (blue arrow) and downsampling (yellow arrow) processes. The decoder network comprises upsampling (green arrow), a feature transformation model (purple arrow), and 3D convolution (red arrow). The upsampling and downsampling blocks share features through skip connections (dashed arrows). Finally, the probability vector is output through the softmax layer. The number next to the feature map indicates the spatial resolution and number of channels of the feature maps.

**Figure 2:** Schematic of the modules in the network. (a) Convolution residual block. (b) Downsampling block and upsampling block. (c) Skip connection. (d) Feature transformation model.

**Figure 3:** Segmentation of critical components. The spring and striker are numbered as 7 and 9, respectively.

**Figure 4:** Three-dimensional rendering of the segmentation results. Sample 1: correct assembly. Sample 2: the striker is assembled to point upward. Sample 3: the spring is assembled below the striker. Sample 4: the spring is assembled below the striker with the striker points upward. Sample 5: the striker is missing. Sample 6: the spring is missing. To avoid occlusion, anatomical diagrams are shown here.

**Figure 5:** Slices of the segmentation results. The yellow, red, and green areas indicate the ground truth, predicted segmentation, and overlap area, respectively. To make the difference prominent, we display magnified views of partial areas, which are marked with red boxes.

**Figure 6:** Segmentation results of the different algorithms.

**Figure 7:** Slices of the segmentation results of the different algorithms. The yellow, red, and green areas indicate the ground truth, predicted segmentation, and overlap area, respectively. To make the difference prominent, we display magnified views of partial areas, which are marked with red boxes.

**Figure 8:** Segmentation results under the different noise levels. The first row shows the projections under the different levels of noise. The second row shows the predicted segmentation results. The zoomed regions of interest are shown on the right side.

**Figure 9:** Segmentation results in different occlusion cases. Case 1: without occlusion. Case 2: with occlusion. Case 3: no striker. The striker is marked with a red box, and the zoomed views are shown on the right side. The grayscale level profiles are extracted along with the red dashed line.

**Figure 10:** Segmentation results of untrained data. Case 1: the striker missed with the spring stuck upside. Case 2: the spring missed with the striker stuck upside.

**Table 1:** Parametric structure of the essential components.

Layer	Parameters	Output size
ResConv block (*k*)	3 × 3 × *k* Conv + BN + ReLU	256^2^ × *k*
	3 × 3 × *k* Conv + BN	
	1 × 1 × *k* Conv	
	ReLU	

DownSample block (*n*)	ResConv block (512)	*n* ^2^ × 512
	ResConv block (512)	
	2 × 2 max-pooling	

UpSample block (*n*)	3 × 3 Deconv with 2 × 2 stride	*n* ^2^ × 512
	ResConv block (512)	
	ResConv block (512)	

Skip connect (*n*)	Concatenate + 1 × 1 × 512 Conv	*n* ^2^ × 512

Transformation module	1 × 1 × 512 Conv + ReLU	256^3^ × 2
	Reshape	
	1 × 1 × 1 × 2 Conv	

3D Conv block (*k*)	3 × 3 × 3 × *k* Conv + BN + ReLU	256^3^ × *k*

*k* denotes the number of filters in the convolution layers, and *n* denotes the output resolution of the downsampling or upsampling block.

**Table 2:** Parametric structure of the entire network.

	Layer	Output size
Encoder network	ResConv block (64)	256^2^ × 64
	ResConv block (128)	256^2^ × 128
	ResConv block (256)	256^2^ × 256
	ResConv block (512)	256^2^ × 512
	DownSample block (128)	128^2^ × 512
	DownSample block (64)	64^2^ × 512
	DownSample block (32)	32^2^ × 512
	DownSample block (16)	16^2^ × 512
	DownSample block (8)	8^2^ × 512

Decoder network	UpSample block (16)	16^2^ × 512
	UpSample block (32)	32^2^ × 512
	UpSample block (64)	64^2^ × 512
	UpSample block (128)	128^2^ × 512
	UpSample block (256)	256^2^ × 512
	Transformation module	256^3^ × 2
	3D Conv block (4)	256^3^ × 4
	3D Conv block (8)	256^3^ × 8
	3D Conv block (16)	256^3^ × 16
	1 × 1 × 1 Conv + softmax	256^3^ × 15

**Table 3:** Quantitative results obtained by the different component segmentations.

Components no.	1	2	3	4	5	6	7
DSC (%)	98.6	97.5	97.6	97.8	97.5	96.7	92.7
JSC (%)	97.3	96.1	97.3	96.6	96.1	94.9	91.6
PPV (%)	97.6	97.0	97.5	97.5	97.5	95.2	91.6
SEN (%)	98.6	98.1	98.7	98.0	97.5	98.5	93.7

Components no.	8	9	10	11	12	13	14
DSC (%)	96.7	91.6	97.2	98.1	97.0	98.6	96.8
JSC (%)	95.6	90.2	96.4	97.4	95.2	97.3	94.8
PPV (%)	95.6	90.8	96.4	97.4	95.2	97.4	94.8
SEN (%)	98.9	92.4	98.8	98.9	98.8	98.8	98.7

**Table 4:** Quantitative results obtained by the different segmentation algorithms.

	V-Net	3D U-Net	Ours
DSC (%)	97.2	96.8	96.7
JSC (%)	96.1	95.7	95.4
PPV (%)	96.2	96.4	95.8
SEN (%)	97.6	97.5	97.7

**Table 5:** Quantitative results obtained under the different noise levels.

	*b*_*0*_ = 1 × 10^5^	*b*_*0*_ = 1 × 10^4^	*b*_*0*_ = 4 × 10^3^
DSC (%)	96.5	96.2	94.8
JSC (%)	95.1	94.6	92.0
PPV (%)	95.6	95.1	93.0
SEN (%)	97.4	97.4	96.7

**Table 6:** Quantitative results obtained by untrained assembly errors.

	Case 1	Case 2
DSC (%)	96.6	96.5
JSC (%)	95.2	95.3
PPV (%)	95.6	95.6
SEN (%)	97.5	97.4

## Data Availability

The data used to support the findings of this study are available from the corresponding author upon request.
